# Gum Acacia Functionalized Colloidal Gold Nanoparticles of Letrozole as Biocompatible Drug Delivery Carrier for Treatment of Breast Cancer

This article has been retracted.

**DOI:** 10.3390/pharmaceutics13101554

**Published:** 2021-09-24

**Authors:** Hibah M. Aldawsari, Sima Singh, Nabil A. Alhakamy, Rana B. Bakhaidar, Abdulrahman A. Halwani, Shaimaa M. Badr-Eldin

**Affiliations:** 1 Department of Pharmaceutics, Faculty of Pharmacy, King Abdulaziz University, Jeddah 21589, Saudi Arabia; nalhakamy@kau.edu.sa (N.A.A.); rbakhaidar@kau.edu.sa (R.B.B.); aahalwani@kau.edu.sa (A.A.H.); 2 Center of Excellence for Drug Research and Pharmaceutical Industries, King Abdulaziz University, Jeddah 21589, Saudi Arabia; 3 IES Institute of Pharmacy, IES University Campus, Bhopal 462044, India; simasingh87@gmail.com; 4 Mohamed Saeed Tamer Chair for Pharmaceutical Industries, Faculty of Pharmacy, King Abdulaziz University, Jeddah 21589, Saudi Arabia

**Keywords:** breast cancer, letrozole, biocompatibility, gold nanoparticles, Gum acacia

## Abstract

The most prevalent malignancy among postmenopausal women is breast cancer. It is one of the leading causes of cancer-related mortality among women. Letrozole (LTZ) is a clinically approved inhibitor for breast cancer in postmenopausal women. However, due to poor aqueous solubility, non-specific binding, unwanted toxicity, and poor blood circulation hampered its clinical applications. To maximize the pharmacological effects and minimize the side effects, inorganic nanoparticles are a good alternative. Due to excellent biocompatibility and minimum cytotoxicity, gold nanoparticles (AuNPs) offer distinct benefits over other metal nanoparticles. Emerging as attractive components, AuNPs and Gum acacia (GA) have been extensively studied as biologically safe nanomaterials for the treatment of cancers. This study reports the synthesis and characterization of GA stabilized gold nanoparticles (GA-AuNPs) of LTZ for breast cancer treatment. The observed particle size of optimized LTZ @ GA-AuNPs was 81.81 ± 4.24 nm in size, 0.286 ± 0.143 of polydispersity index (PDI) and −14.6 ± −0.73 mV zeta potential. The biologically synthesized LTZ @ GA-AuNPs also demonstrated dose-dependent cytotoxicity against the human breast cancer cell line MCF-7, with an inhibitory concentration (IC_50_) of 3.217 ± 0.247. We determined the hemolytic properties of the LTZ @ GA-AuNPs to evaluate the interaction between the nanoparticles and blood components. Results showed that there is no interaction between LTZ @ GA-AuNPs and blood. In conclusion, the findings indicate that LTZ @ GA-AuNPs has significant potential as a promising drug delivery carrier for treating breast cancer in postmenopausal women.

## 1. Introduction

Breast cancer, in its advanced stages, is one of the leading causes of cancer-related fatalities in women worldwide, mainly in the United States [1,2]. Most breast cancers are estrogen receptor-positive (ER+) and human epidermal growth factor receptor 2 (HER2)-negative tumors [3]. Because of the expression of estrogen receptor alpha (ERα), most breast cancer cases are classified as ER+; such patients have a 5-year overall survival rate of almost 90% [4,5]. The presence or absence of the targetable biomarkers ER, progesterone receptor (PgR), and HER2 determines the course of breast cancer treatment in such individuals. It has been recommended that endocrine therapy be used first in treating females with ER+ advanced-stage breast cancer rather than chemotherapy, except in the event of rapidly progressing illness [6,7]. Antiestrogens, selective estrogen receptor modulators (SERMS), selective estrogen receptor degraders (SERDs), and aromatase inhibitors (AIs) are being used to prevent estrogen from binding to the ER [8,9].

Letrozole (LTZ) is an orally available third-generation aromatase inhibitor that works as an efficient non-steroidal anticancer drug [10]. The fact that it can block excessive estrogen production means it is referred to as an estrogen receptor-positive breast cancer therapy [11]. Compared to tamoxifen, the medication has comparatively good efficacy and safety profile. The Food and Drug Administration (FDA) has approved adjuvant chemotherapy to treat hormone-positive or metastatic breast tumors in postmenopausal women that have spread to other areas of the body [12,13,14]. Clinical trial investigations have shown that it inhibits peripheral aromatase by more than 98%. After only two weeks of therapy, it reduces blood and urine estrogen levels by more than 95% in postmenopausal women [15].

The half-life of LTZ is two days, and its plasma concentrations reach a steady state in an average of 2 to 6 weeks after being administered [16]. Although these concentrations are 1.5–2 times greater than the predicted values, this indicates a nonlinear pharmacokinetic release profile [17]. The therapeutic window of the drug is exceeded because of this non-linearity in the drug release profile, resulting in significant side effects. In this instance, however, the current therapeutic options are primarily palliative, and the development of resistance to therapies is a frequent occurrence [18]. As a result, it is critical to prevent this phenomenon by developing novel delivery methods with correctly anticipated pharmacokinetics, allowing LTZ to remain within therapeutic levels.

Meanwhile, researchers are searching for vehicles that would deliver drugs precisely to the targeted organ or tissue. A delivery mechanism that can permeate both the cellular and outer mitochondrial membranes is being developed by scientists to induce apoptosis more efficiently and effectively. The targeted drug delivery system based on nanoparticles has gained considerable attention in cancer treatment during the last few decades [19,20,21]. Inorganic nanoparticles have attracted a significant deal of attention in recent years due to several advantages and distinguishing characteristics that they offer, notably in imaging and drug delivery. For nanomedicine, the growth of an extensive range of NPs with the versatility to alter size, composition, and functioning during the previous several decades has advanced this technology [22].

Gold nanoparticles (AuNPs; authorized by the FDA) are among the most widely utilized inorganic nanoparticles in biomedical applications because of their excellent compatibility with the biological system, small size, reduced toxicity, simplicity of surface tailoring, and controlled drug release properties [23]. Although AuNPs are effective in cancer treatment, they are subsequently removed by the reticular endothelium system, particularly macrophages, restricting their use. To bypass this constraint, the shape and surface chemistry of AuNPs can be modified by their fabrication method. AuNPs are synthesized and functionalized in a variety of ways using different techniques. The traditional methods for the fabrication of AuNPs are based on reducing agents such as sodium borohydride, trisodium citrate, and other similar compounds. However, the toxicity of these reducing agents, as well as the presence of organic solvents, are significant limits [24].

The need for nontoxic and biocompatible AuNPs with small particle size, aggregation prevention, and the ability to introduce functionality to the particle surface for the conjugation of biomolecules has thus been identified. The search is currently underway for a one-step solution to all of these issues. The utilization of natural materials such as natural polysaccharides and gums might help to overcome this constraint.

In the present study, an attempt has been made to synthesize AuNPs by utilizing Gum acacia (GA). GA is a naturally occurring polysaccharide with a branching structure with slightly acidic. The major structural components present in GA include α-l-rhamnopyranosyl, β-d-glucuronopyranosyl, and 4-O-methyl-β-d-glucuronopyranosyl, α-l-arabinofuranosyl units [25,26]. This research aimed to synthesize ecologically friendly LTZ capped gold nanoparticles by employing GA as a reducing agent for breast cancer treatment. To our knowledge, this is the first to report on the synthesis and characterization of LTZ formulations based on the usage of GA-AuNPs.

## 2. Materials and Methods

### 2.1. Materials

Gold chloride (HAuCl_4_·3H_2_O) (Sigma-Aldrich) was utilized without additional purification. LobaChemie Laboratory Reagents & Fine Chemicals Pvt. Ltd. (Mumbai, India) provided the medium molecular weight GA used in this study. Letrozole powder (HPLC grade 99.12%) was kindly gifted by Hetero drugs Pvt. Ltd. (Hyderabad, India). Di-sodium hydrogen phosphate dihydrate (Na_2_HPO_4_·2H_2_O) (Sigma-Aldrich, St. Louis, MO, USA) and Sodium dihydrogen orthophosphate dihydrate (NaH_2_PO_4_·2H_2_O) (Merck, Kenilworth, NJ, USA) were used to prepare 0.1 M phosphate buffer solution (PBS). The pH of PB was adjusted by adding Ortho Phosphoric acid (H_3_PO_4_).

Dimethylsulfoxide (DMSO), Dulbecco’s modified Eagle’s medium (DMEM), MTT [3-(4,5-dimethylthiazol-2-yl)-2,5-diphenyl tetrazolium bromide], trypsin, EDTA, and phosphate-buffered saline (PBS) were purchased from Sigma Chemicals. Fetal bovine serum (FBS) was purchased from Gibco. Flasks (25 and 75 cm^2^) and 96-well plates were purchased from Eppendorf, India. MCF-7 cell lines were purchased from NCCS, Pune. The cells were maintained in MEM supplemented with 10% FBS and penicillin/streptomycin (0.5 mL^−1^) in an atmosphere of 5% CO_2_/95% air at 37 °C. All aqueous solutions were made with ultra-high purity water filtered with Mill-Q Plus equipment (Millipore Co., Burlington, MA, USA). Analytical grade solvents and chemicals were used in their purest form and were not further purified.

### 2.2. Preparation of Gum Acacia Solution

Firstly, Gum acacia (GA) was powdered and filtered through a sieve with a mesh size of 250. A combination of Milli-Q water and ethanol in a 1:1 ratio was used to make a stock solution of 1% *w*/*v* gum. The solution was left to stir for 30 min at ambient temperature. The product was centrifuged at 10,000 rpm for 30 min, and the supernatant was decanted to separate the final GA solution. The supernatant produced was collected, air-dried, and then utilized in the experiment.

### 2.3. Preparation of Gold Chloride Solution

To obtain the gold chloride solution, 3.96 mg of gold chloride (HAuCl_4_·3H_2_O) was dissolved in 0.25 mL Milli-Q water and 0.25 mL ethanol. It was kept for solubilization using a magnetic stirrer for 15 min.

### 2.4. Synthesis of Gold Nanoparticles (AuNPs)

Stabilized colloidal AuNPs were synthesized according to a previously described method, with slide modification [27]. For synthesis, 100 mL of HAuCl_4_ solution (10 mM) was added to 5 mL of GA solution (1% *w*/*v*). Then, the temperature was maintained at 80 ± 1 °C with continual stirring for an additional 30 min. One hour after the start of the experiment, a dramatic shift in color from colorless to ruby red could be noticed. This served as proof of the synthesis of AuNPs.

### 2.5. UV–Visible Spectroscopy

The synthesized GA-AuNPs were confirmed by UV–Vis spectroscopy with slight modification to the method given by Nakamura et al. [28]. Three milliliters of a gold aqueous solution was placed in a quartz glass cuvette that was optically transparent at the incident laser wavelength. The laser beam was supplied into the cuvette and fully focused on the solution using an aspherical lens.

### 2.6. Drug Capping

LTZ was slightly soluble in ethanol. To make it completely soluble, we added DI water and ethanol at a 1:1 ratio. The solution was stirred for 15–20 min. After stirring for 20 min, 15 mL of GA-AuNPs was added to this solution with continuous stirring at room temperature for 24 h. No precipitation of the drug was observed. It was further centrifuged at 15,000 rpm for 30 min. LTZ-encapsulated GA stabilized colloidal gold nanoparticles were collected for further study. The drug content in the supernatant was determined using UV–Vis absorption spectroscopy (Shimadzu UV 1601, Kyoto, Japan) at 240 nm. The % drug capping was established by Equation (1):

(1) $$\%\;\mathrm{Drug}\;\mathrm{capped}=\frac{\left(Total\;amount\;of\;LTZ\;added-Amount\;of\;free\;LTZ\;in\;supernatent\right)}{Total\;amount\;of\;LTZ\;added}\times 100$$

### 2.7. Characterization of Nanoparticles

#### 2.7.1. Hydrodynamic Diameter and Surface Charges Measurement

Dynamic light scattering (DLS) was applied for size determination. Malvern Zetasizer Nano ZS (Model S, Ver. 2.15, Malvern Panalytical, Malvern, UK) was used to measure the mean diameter, polydispersity index (PDI), and zeta potential (ZP) of LTZ-GA-AuNPs. The hydrodynamic diameter was evaluated after suspending the prepared colloidal nanoparticles in deionized water. The extent of DLS was prepared through a laser wavelength of 633.0 nm at 25 °C by a revealing angle of 90°. All samples were analyzed in triplicate and the three cycles were averaged.

#### 2.7.2. Fourier Transform Infrared Analysis

Individual samples of either LTZ or LTZ-GA-AuNPs were combined with KBr and then compressed into a pellet using a hydraulic press. The resulting pellets were examined using an FTIR spectrophotometer (Spectrum BX, Perkin Elmer, Waltham, MA, USA) in the range of 4000–400 cm^−1^.

#### 2.7.3. Morphology Study

Field emission scanning electron microscopy (FE-SEM) (Supra 55, Carl Zeiss, Jena, Germany) was used for observing the morphology of the LTZ-GA-AuNPs. It was equipped with a tungsten filament, which covers the sample, gives high-quality pictures with minute electrical impulses, and has an advantage over high-resolution transmission electron microscopy (HR-TEM).

HR-TEM and selected area electron diffraction (SAED) (JEOL 2100 HRTEM, Seoul, Korea) were used for the morphology study. For this, a drop of the sample was drop cast on a carbon-coated copper grid. It was then air-dried at room temperature and stained with 2% uranyl acetate.

#### 2.7.4. In Vitro Release Studies

As previously reported, in vitro LTZ release from LTZ-GA-AuNPs was evaluated using the dialysis bag technique in phosphate-buffered saline (PBS; pH 7.4) and simulated cancerous conditions (pH 5.0) in vitro for 72 h, at 37 °C, respectively. The dialysis membrane used has a molecular weight cut-off (MWCO) between 12,000 to 14,000 Da. A sample of LTZ-GA-AuNPs equivalent to 5 mg of LTZ was dissolved in 5 mL of distilled water and sealed in a dialysis bag. Five hundred milliliters of either PBS pH 7.4 or sodium acetate buffer pH 5.0 was used as a release medium. Samples of 5 mL were withdrawn at regular time intervals for 72 h and replaced with an equivalent volume of fresh medium. The samples were quantified for the released drug by UV spectrophotometer at 240.00 nm.

#### 2.7.5. In Vitro Hemolysis Assay

The use of blood hemolysis tests determined the biocompatibility of the nanocarriers. A minor modification to the previously published procedure technique was performed [29]. LTZ-GA-AuNPs and LTZ were tested for hemolytic activity at a dose of 1 mg/mL. Male Wistar rat serum (5 mL) was drawn from a closed bottle of Ethylenediaminetetraacetic acid (EDTA) glazed tube and utilized within an hour. Blood was centrifuged at 3000 rpm for 10 min to separate red blood cells (RBCs) from the blood samples. Separated RBCs remained eroded three times by PBS (7.4) and diluted through 900 μg of the saline solution for the negative control and with 1% Triton X-100 for the positive control. A round-bottom 96-well plate containing RBCs suspension (100 μL) was treated with different concentrations of nanocarriers. Finally, the plate was stirred lightly and further incubated for 3 h at 37 °C. The obtained supernatant was determined by a UV–Vis spectrophotometer via a plate reader at 541 nm. The percentage of hemolysis was calculated by Equation (2), where *At* is the absorbance of the treated supernatant, *Ac* is the absorbance of the negative control, and *Ax* is the absorbance of the positive control [30].

(2) $$\%\;\mathrm{Hemolysis}=\frac{\left(At-Ac\right)}{\left(Ax-Ac\right)}\times 100$$

#### 2.7.6. In Vitro Anticancer Activity by MTT Assay

The cell viability in the Human breast cancer cell line (MCF-7) was determined by the MTT assay as previously described [24,25]. The cells were cultured and scattered in 96-well cell culture plates (Greiner CELLSTAR^®^ 96-well plates, Merck) at a 2 × 10^6^ cells/well concentration. Different concentrations of LTZ and LTZ-GA-AuNPs were added to the wells seeded with cells. The plates were incubated for 48 h. Consequently, the sample-laden medium was replaced with 100 μL of fresh culture medium and 20 μL of MTT solution (5 mg/mL in PBS) in each corresponding well. An aliquot (85 μL) from the wells was removed, and 50 μL of DMSO from each well was added and wholly mixed with the pipette and further incubated at 37 °C for 10 min. From the microplate reader (Spectrostar Nano, BMG Labtech, Ortenberg, Germany), cell viability was determined at 540 nm, which is based on the ability of viable cells to decrease the tetrazolium component of MTT into purple-colored formazan crystals [31]

The % cell viability was calculated by Equation (3).

% Cell viability = ((A540 nm treated cells))/((A540 nm untreated cells)) × 100(3)

The IC_50_ value was determined by using a linear regression equation, i.e., y = mx + c.

Here, y = 50, m, and c values were derived from the viability graph. A value of *p* < 0.05 was considered statistically significant.

#### 2.7.7. Stability Studies

A short-term physical stability revision was maintained to govern the influence of temperature on LTZ-GA-AuNPs. The stability of LTZ-GA-AuNPs was examined at temperatures of 25 ± 1 °C for 30 days. The mean particle size, polydispersity, and zeta potential of LTZ-GA-AuNPs were measured to assess physical stability [32].

## 3. Results and Discussion

### 3.1. Chemical Characterization Letrozole-Loaded GA-AuNPs

In the current work, we synthesized LTZ-encapsulated GA-AuNPs by reducing a charged gold atom (Au^3+^) to a neutral gold atom (Au^0^). GA was used as a reducing and capping agent in this experiment. Many variables, including temperature, reaction time, gum concentration, gold concentration, and the gold-to-gum ratio, were observed to influence the synthesis of gold nanoparticles in the study. The overall synthetic method did not use any toxic chemical reagents. The color of the gold solution did not change until it reached a temperature of 50 °C. At 60 °C, the color of the solution changed from colorless to violet due to a further increase in temperature as shown in Figure 1a,b. As illustrated in Figure 1e, the formation of AuNPs may be seen as a shift in color to red-violet. The surface plasmon resonance (SPR) of AuNPs, which is linked to the oscillation of free conducting electrons generated by the electromagnetic field, was responsible for the reddish-violet color seen [33]. Further confirmation of the formation of the nanoparticles in the aqueous solution was carried out by UV–Vis spectroscopy. The solution was scanned within a range of 200–800 nm. The maximum absorbance was recorded at a wavelength of 280 nm. During the first hour of incubation, the intensity of the absorption peak increased significantly. The incubation period of Letrozole-loaded GA-AuNPs (1 h, 2 h, and 3 h) did not result in a significant rise in the intensity of the SPR band after an additional hour of incubation time. As illustrated in Figure 1c, it denotes the completion of a reaction after one hour of incubation. The results indicated that the reaction time did not affect the absorbance wavelength. Based on the findings, it was determined that the reaction time had no effect on the absorbance wavelength.

### 3.2. Fourier Transform Infrared Analysis

To further understand the potential functional groups involved in the characterization of Letrozole-loaded GA-AuNPs, Fourier transform infrared spectroscopy (FTIR) was used, as shown in Figure 1d. The characteristic bands of AuNPs, relative to the symmetric and asymmetric stretching vibrations of –CH_2_ at 2918 and 2850 cm^−1^, were maintained in the GA-AuNPs. The symmetric stretching vibration frequency of OH observed at 3363 cm^−1^ indicated the presence of alcohols, which proves the bonding between metal and carboxylic oxygen according to the previous study [34]. The secondary alcohol group (C–O) peaked at 1015.094 cm^−1^. The structural characteristics found in the FTIR analysis were in excellent agreement with the data obtained from UV, indicating that the crystalline Letrozole-loaded GA-AuNPs were synthesized.

### 3.3. Shape, Particle Size, Polydispersity Index, and Zeta Potential

Following the preparation, LTZ @ GA-AuNPs were characterized for their morphological features. The characters of AuNPs depend on morphological features such as the appearance and crystal characteristics of nanoparticles. The morphological examination was carried out using field emission scanning electron microscopy (FE-SEM) and high-resolution transmission electron microscopy (HRTEM). FE-SEM of the air-dried LTZ @ GA-AuNPs mainly showed spherical in shape, as shown in Figure 2a. Non-spherical particles are in uniform shapes and sizes depending on the angle from which they are observed.

Nanoparticle shape and surface morphology were also investigated by HR-TEM analysis. Figure 2b shows the HR-TEM images of the lyophilized LTZ @ GA-AuNPs. HR-TEM images are in alignment with FE-SEM images. It demonstrates that the LTZ @ GA-AuNPs were spherical in shape. The nanoparticles prepared were spherical, had uniform particle size, and had a smooth surface on the surface. It can be observed that all of the AuNPs have icosahedral structures that are identical to one another. All are monodispersed with a mean diameter of around 100 nm. Although there are some overlaps between sections of gold nanoparticles, they are not agglomerated; rather, each particle’s shape remains preserved.

Figure 2c depicts the crystalline nature of LTZ-GA-AuNPs, which was also confirmed by SAED. In this research, we observed that brilliant circular pattern rings were detected in a circular pattern. This might reflect the lattice planes of crystalline Au nanoparticles, which would explain their appearance. This finding was found to be somewhat associated with the HR-TEM results. This result was in support of previously published work [27].

We performed dynamic light scattering (DLS) to quantify the size distributions, polydispersity index (PDI), and zeta sizer to further understand these characteristics. According to Figure 2d, the average size of blank and loaded nanoparticles was 50 nm and 81.8 nm, respectively, showing a relative size enlargement upon LTZ loading. DLS analysis revealed a mean particle size of 81.81 ± 4.24 nm in size, 0.286 ± 0.143 0.286 PDI for the prepared LTZ-GA-AuNPs, indicating high monodispersity of nanoparticles (Figure 2d. The colloidal stability of nanoparticles was explored by determining the magnitude of their surface charges. The surface charge of NPs remains a significant constraint such regulates bioavailability and lifetime [35]. The zeta potential of the synthesized nanoparticles was −14.6 ± 0.73 mV at pH 7, as shown in Figure 2e. Because of the high molecular weight and the significant number of free hydroxyl groups in the structure of GA, the Au nanoparticles were negatively charged [36]. The measured zeta potential values suggested that the nanoparticles became more anionic after LTZ loading. The negative charge indicated accurate surface charge for extensive half-lives and great biodistribution and ensured the stability of the nanocomposite in biological environments, allowing target sites [37].

### 3.4. Drug Capping

A prospective drug carrier needs to have a high loading capacity as well as structural integrity. As a result, it is critical to investigate the maximum drug loading as well as relative conditions. Therefore, the capping of LTZ by GA-AuNPs was tested to assess their potential use as nanovectors in this context. The drug capping was found to be 42%.

### 3.5. In Vitro Drug Release

LTZ was chosen as a cancer model drug for breast cancer. As shown in Figure 3, we studied the drug release of LTZ @ GA-AuNPs at different pH conditions. The release behavior of the LTZ @ GA-AuNPs was examined to determine whether they are capable of performing controlled release in physiological conditions or not when used as drug carriers. To assess drug release characteristics, the LTZ-loaded GA-AuNPs were suspended in phosphate buffer solutions with pH values of 5 and 7.4 at 37 °C. These conditions are close to a cancer cell’s physiological and endosomal pH conditions, respectively, as shown in Figure 3. The drug was released from LTZ @ GA-AuNPs in PBS (pH 7.4). The time-dependent accumulated drug release (ADR) curves displayed a prolonged release profile with no noticeable burst effect at pH 5 and 7.4. The prolonged-release rate would yield a steady-state drug concentration and provide adequate time for LTZ @GA-AuNPs to build up at the tumor site. Further, as shown in Figure 3, the % LTZ released over 72 h was about 80.5% at pH 7.4 and 91.5% at pH 5, indicating the sensitivity of the LTZ-GA-AuNPs to the endosomal pH values of a cancer cell environment. As a result, LTZ was released faster under acidic conditions (pH 5.0, 37 °C) than physiologic conditions (pH 7.4, 37 °C). Previous studies also reported a greater % of drug released from GA-AuNPs in acidic conditions compared to neutral conditions [27]. LTZ @ GA-AuNPs nanosystem was more easily released under acidic conditions than it was under neutral pH, which is advantageous in reducing the toxicity of LTZ on normal tissue, as evidenced by these results. According to these findings, the decreased pH in cancer cells stimulated the release of LTZ from LTZ @ GA-AuNPs. To accomplish LTZ drug release, LTZ @ GA-AuNPs may first enter the cytoplasm and aggregate in lysosomes (pH 4.5–5.0), after which the drug enters the nucleus [38,39].

### 3.6. In Vitro Hemolysis Assay

Hemolytic toxicity of GA stabilized gold nanoparticles was examined against RBC suspension (2% hematocrit). As a standard hemolytic agent, Triton X-100 (1% *v*/*v*) was utilized, and the absorbance value of Triton X-100 was regarded to signify total (100%) hemolysis. Triton is a nonionic surfactant that causes the rupture of the RBC membrane, resulting in the release of hemoglobin. Figure 4a shows the results of the influence of gold nanoparticles on hemolysis at various concentrations (5–20 g/mL). GA-AuNPs displayed significantly less hemolysis (2%). The hemolysis effects of LTZ-GA-AuNPs at concentrations of 5, 10, 15, and 20 µg mL^−1^ were consistent with the limits of less than 15%. Furthermore, as AuNPs are biocompatible and non-toxic, they are considered to be superior drug delivery vehicles. The above studies on RBCs suggest that the synthesized LTZ-GA-AuNPs in the present study are potentially biocompatible and safely used inside the body.

### 3.7. MTT Assay

The results of the MTT test, which measures cell viability, provide unambiguous explanations for the methods used by cells to respond to a toxic substance. In the present study, the synthesized LTZ-GA-AuNPs showed a higher anticancer activity to the MCF-7 breast cancer cell line than LTZ, with dose-dependent cellular toxicity. LTZ-GA-AuNPs showed good cytotoxic activity against the breast cancer cells in a concentration-dependent manner. In line with this, our findings suggest that LTZ can be employed in treating breast cancer since it showed higher cytotoxic effects to tumor cells when it was conjugated to GA-AuNPs, as shown in Figure 4b and Figure 5. The IC_50_ value of LTZ-GA-AuNPs was 3.217 ± 0.247 µg.

### 3.8. Stability Studies

The novel LTZ @ GA-AuNPs formulation was studied for its stability for one month at room temperature (RT) as shown in Table 1. The size of the particle, % drug capped, PDI, and zeta potential (*p* > 0.5) were observed to be negligible. Based on the stability study, it can be concluded that the newly synthesized formulation is stable and can direct the exploration of applications in targeted drug delivery therapy.

## 4. Conclusions

Breast cancer in postmenopausal women is one of the leading causes of cancer-related deaths in women. The recent promising applicability of Letrozole (LTZ) as an anticancer drug has been approved for breast cancer treatment in postmenopausal women. However, this therapy has appreciable side effects. Nanoscale carriers, such as metal nanoparticles and polysaccharides, are being widely utilized as drug delivery vehicles to target tumor cells precisely. Biologically inspired green synthesis of nanoparticles has become a promising alternative against the chemically fabricated process considering reduced toxicity. This work introduced a new approach for breast cancer therapy using LTZ-GA-AuNPs as LTZ delivery. This study reports a safe and rapid method for the green synthesis and characterization of GA-AuNPs. The structural and morphological properties are confirmed by SEM and HR-TEM, respectively. Material characterizations confirmed the uniform LTZ within GA-AuNPs in the size range of 81.81 nm, 0.286 of PDI, and −14.6 mV zeta potential. The in vitro cytotoxicity with LTZ-GA-AuNPs showed better therapeutic efficacy than bare LTZ in the MCF-7 cell line. Thus, the LTZ-GA-AuNPs-based drug delivery system provided a reliable therapeutic strategy for treating breast cancer.

## Figures and Tables

**Figure 1:** Characterization and chemical structure of LTZ@ GA-AuNPs: (**a**,**b**) Formation of optimized GA stabilized gold nanoparticles (GA-AuNPs) under natural light in transparent glass; (**c**) UV study of Letrozole-loaded GA-AuNPs; (**d**) Comparative FTIR spectra of drug and drug-Au; (**e**) final optimized formulation.

**Figure 2:** Characterization of LTZ@ GA-AuNPs (**a**) FE-SEM image; (**b**) HR-TEM image; (**c**) SAED; (**d**) DLS exemplifying the size distribution of the particles formed; (**e**) zeta potential.

**Figure 3:** In vitro cumulative percentage drug release study of LTZ @ GA-AuNPs pH = 5 and 7.4 at 37 °C.

**Figure 4:** (**a**) In vitro hemolysis percentage of LTZ-GA-AuNPs; (**b**) in vitro cytotoxicity and percent cell viability assay against MCF-7.

**Figure 5:** Morphological changes of the human breast cancer cell line MCF-7 after given treatment; (**a**) control; (**b**) 1 µg; (**c**) 5 µg; (**d**) 10 µg; (**e**) 15 µg; (**f**) 20 µg.

**Table 1:** Effect of storage conditions at ambient temperature (25 °C) and time (days) on size, PDI, ZP (mV), and % drug capped of LTZ @ GA-AuNPs.

Time (Days)	Size (nm)	PDI	ZP (mV)	% Drug Capped
0	81.81 ± 4.0905	0.286 ± 0.143	−14.6 ± −0.73	40 ± 2
7	81.93 ± 4.0965	0.279 ± 0.01395	−14.4 ± −0.72	41 ± 2.05
15	81.99 ± 4.0995	0.289 ± 0.01445	−14.6 ± −0.73	40 ± 2
30	82.95 ± 4.1475	0.298 ± 0.0149	−14.7 ± −0.73	40.2 ± 2.01

All experimental result values are expressed as the mean ± SD (*n* = 3).

## Data Availability

The data presented in this study are available on request from the corresponding author.
